RETRACTED

# Quantitative analysis and visualization of literature on acupuncture and related TCM therapies for the treatment of colorectal cancer based on CiteSpace

**DOI:** 10.3389/fonc.2023.1290588

**Published:** 2024-01-05

**Authors:** Zeli Li, Qianwen Xiong, Shuwen Li, Wenxiang Chen, Nenggui Xu, Fanghua Qiu

**Affiliations:** ^1^ Clinical Medical College of Acu-Moxi and Rehabilitation, South China Research Center for Acupuncture and Moxibustion, Guangzhou University of Chinese Medicine, Guangzhou, China; ^2^ Guangzhou University of Chinese Medicine, Guangzhou, China; ^3^ The Affiliated TCM Hospital of Guangzhou Medical University, Guangzhou, China; ^4^ Department of Infection Control, Guangzhou Hospital of Traditional Chinese Medicine, Guangzhou, China

**Keywords:** acupuncture, colorectal cancer, Citespace, literature measurement, visualization analysis

## Abstract

**Objective:**

We analyzed the literature describing the results of treatment of colorectal cancer (CRC) using acupuncture in the past three decades from the Web of Science (WoS) and Chinese databases (including CNKI, WANGFANG and VIP), and summarized the current development of CRC treatment as well as future research directions through the presentation of maps and visualization analysis.

**Methods:**

We searched the WoS and Chinese databases. Relevant articles were exported, and the data were organized using Excel software and was visualized and analyzed using CiteSpace software.

**Results:**

A total of 355 articles from the WoS and 95 articles from Chinese databases were selected for inclusion in the analysis. The articles in WoS were sourced from 174 journals, 1274 institutions, and 66 countries, and covered 299 keywords. The articles in the Chinese databases were sourced from 43 journals, 111 institutions, and 3 countries, and included 126 keywords. The article with the most citations in the WoS was cited 128 times and in the Chinese databases, the article with the most citations was cited 120 times. Acupuncture, CRC, rectal cancer, apoptosis, warm acupuncture, traditional Chinese medicine (TCM) and gastrointestinal function were mentioned most frequently in the WoS. CRC, electroacupuncture, gastrointestinal function, rectal cancer, acupuncture and moxibustion, acupuncture, and colon cancer were mentioned most frequently in the Chinese databases.

**Conclusion:**

Both the WoS and Chinese databases showed a gradual increase in the number of articles related to acupuncture treatment for CRC, indicating a growing interest in this area. Acupuncture treatments are diverse, including warm acupuncture, auricular acupuncture, acupuncture injection, and electroacupuncture. They are often used in combination with drugs to treat symptoms such as depression, nausea and vomiting, pain, diarrhea, and urinary and fecal incontinence, which are commonly associated with CRC.

RETRACTED

## 1 Introduction

The number of patients with colorectal cancer (CRC) has been increasing throughout the world in recent years, and most are diagnosed at advanced stages with very high mortality rates (1). As of 2020, CRC has the third highest incidence rate at 10% and the second highest mortality rate at 9.4% worldwide (2). The incidence and number of CRC-related deaths in the world is increasing with age, and the number of patients age <35 is relatively small. After the ages of 40 to 44, the number of patients increases significantly. Less than 20% of patients aged 40 to 44 years can be treated with radical excision and the 5-year survival rate of patients with lung metastases of CRC that cannot be treated with radical surgery is <20% and still has a poor prognosis (3). The rapid increase in the incidence and mortality of CRC and the resulting disease burden have become a main public health concern. Current clinical treatment of CRC is mainly based on surgical treatment, supplemented by systemic chemotherapy, radiotherapy, targeted therapy, and other integrated symptomatic supportive treatment. Meanwhile, during the treatment of patients with CRC, complications from surgery, drug side effects, and the high cost of treatment can result in poor patient adherence. This can lead to difficulties in treatment and even psychological barriers, physiological rejection, and other negative impacts, ultimately reducing the effectiveness of clinical treatment. Medical expenses are high, which brings a heavy economic burden to the patient’s family and society. As a result, CRC has become a pressing global health concern.

As a traditional Chinese nonpharmacological therapy and an alternative therapy for gastrointestinal disease, acupuncture has been used for postoperative treatment and recuperation in recent years and has achieved good results (4). The core idea of acupuncture in the treatment of human diseases is to regulate the physiological functions of the body at distant sites by stimulating specific regions of the body regions (acupoints) (5). Based on the theory of TCM, acupuncture is the process of inserting fine metal needles through the skin and into specific locations along the path of special catheters believed to be electrical signals to stimulate and has the ability to clear the meridians and regulate qi and blood flow, achieving the goal of promoting positive energy and dispelling negative energy (6). Acupuncture has the advantages of high reliability, low toxicity, minimal side effects, and low cost, which can alleviate economic pressure on patients. When combined with traditional Chinese and Western medicine, acupuncture has shown significant advantages in the treatment of CRC. Currently, numerous high-quality clinical studies on acupuncture have greatly increased its acceptance and international influence in the medical field (7). Meanwhile, acupuncture has received increasing attention and the number of related reports has increased year by year, but it still needs a clearer and more scientific generalization and integration system, so that it can be used for clinical promotion.

RETRACTED

CiteSpace is a visual citation analysis software for scientific literature, and has been used to identify and present new trends and developments in scientific development to provide an overview of a research field and to highlight particular important documents in the history of the field’s development (8). The technology of information visualization and knowledge mapping can effectively uncover the research hotspots and frontiers in various fields, including medicine. By presenting the intrinsic connections and hidden information of medical research in the form of visual knowledge maps, this technology provides researchers with new ways to comprehend the latest trends and developments in the medical field. This makes it an invaluable tool for gaining insight and keeping up-to-date with the latest advancements (9). In this study, we utilized CiteSpace to visualize and analyze the selected literature from the WoS. This allowed us to obtain a relevant knowledge map and to clearly and scientifically demonstrate the current development of acupuncture in the treatment of CRC. Our findings lay the foundation for future research experiments.

## 2 Materials and methods

### 2.1 Documentation sources

All articles used in the project were sourced from the WoS and Chinese databases.

### 2.2 Retrieval methods

The subject words were acupuncture and CRC. The search strategy for the WoS was as follows: (SU = ‘acupuncture’ OR ‘auricular acupuncture’ OR ‘acupuncture point buried needle’ OR ‘warm acupuncture’ OR ‘Chinese medicine’ + ‘colon cancer’ OR ‘rectal cancer’ OR ‘intestinal cancer’). Search strategy of CNKI: “SU=(needle + electric + puncture + electric acupuncture + electrical stimulation)*(colorectal cancer + colon cancer + rectal cancer + colorectal cancer)”. Search strategy of Wanfang Data: “Subject:(Needle or electricity or puncture or electroacupuncture or electrical stimulation) AND subject:(Colorectal cancer or colon cancer or colorectal cancer)”. Search strategy of VIP: “M=(needle + electric + puncture + electroacupuncture + electrical stimulation)*(colorectal Cancer + colon cancer + rectal cancer + colorectal cancer)”.

RETRACTED

A total of 507 articles were retrieved from WoS, of which 152 were excluded after careful reading, evaluation, and filtering. The remaining 355 articles were included in the study. In the Chinese databases, 154 articles were retrieved. After careful reading, evaluation, and filtering, 59 articles without direct relevance were excluded, leaving a total of 95 articles included for analysis.

### 2.3 Document conversion

The literature to be analyzed was imported into CiteSpace (v.6.1.R3) in the form of Refworks, the parameters were adjusted, the time interval was selected as January 1993 to July 2023, the year time slice was selected as 1, and the node type was selected as authors, institutions, and keywords, to obtain different types of visualization maps, respectively. Subsequently, the keywords were analyzed by clustering analysis and emergent word analysis.

## 3 Results

We analyzed the number of publications, authors, institutions, and keywords to research acupuncture or combined with other TCM treatments for CRC. We found that research on this topic has increased worldwide in the past 30 years. In this project, we utilized CiteSpace software to gain a more intuitive and clear understanding of the connections and information within the literature. This allowed us to identify the development of hotspots and to provide ideas and directions for future research (10).

### 3.1 Trends in annual literature issuance

Globally, the literature on acupuncture for CRC can be traced back to 1993 at the earliest; which was a reprint of an article originally published in *the Japanese Journal of Oriental Medicine* in 1990 (11). The article describes a clinical study on the use of electroacupuncture to treat postoperative dysuria in patients with rectal cancer. The study demonstrated the effectiveness of electroacupuncture in treating postoperative dysuria. However, there were few publications on this topic in both the WoS and Chinese databases between 2004 and 2012. This could be attributed to the high incidence and mortality rate of CRC, as well as the limited popularity and recognition of acupuncture during that time. The number of publications from the WoS retrieved experienced a surge in 2013, reaching 13, and then remained stable for 5 years. Another surge occurred in 2019, with the number of relevant publications doubling immediately.

Similar to the trend in the WoS database, the number of relevant articles in the Chinese databases increased from 2013 to 2018 and then stabilized. However, the number of relevant articles in Chinese began to increase after 2019, with a peak of 55 articles in 2022. Generally speaking, there has been an increasing number of research papers on acupuncture and other TCM therapies for the treatment of CRC. This suggests that the use of acupuncture or a combination of other TCM therapies to treat CRC is gaining attention in the research community (**Figure 1A**; **Supplementary Table 1**).

RETRACTED

**Figure 1:** Trends in the count of articles from WoS and Chinese databases and author, country and institution visualization and analysis mapping from WoS. **(A)**. The number of publications in WoS and Chinese databases per year; **(B)**. The visual analysis of authors in WoS; **(C)**. The visual analysis of countries in WoS; **(D)**. The visual analysis of institutions in WoS.

### 3.2 Author visual analytics

In the graph, each author is represented by a node, with the font size indicating the number of publications and the number of lines connected to it indicating the level of collaboration. The literature from the WoS includes a total of 2260 authors. Li Qi, Wang Yan, and Chen Youqin have published the most articles. Li Qi has published nine articles with 15 co-authors, including Sui Hua, Jia Ru, and Wang Yan. Chen Youqin has published seven articles and is related to 10 authors (**Figure 1B**; **Supplementary Table 2**). A total of 202 authors of the literature were from the Chinese databases. MENG Jinhai, MAI Sicong, and GU Meiying published the most articles (**Supplementary Table 2**). Despite the extensive and widespread collaboration network, there is currently no large-scale joint collaboration system in place, and cross-team collaboration is nonexistent.

### 3.3 Countries and institutional distribution analysis

Each country or institution is represented by a node, and a line connecting countries or institutions indicates their affiliation or cooperation. The font size of each node reflects the level of activity of the country’s or institution’s articles. We analyzed the collaborative network maps of each country in the WoS literature and obtained the number of publications from the top 10 countries (**Figure 1C**). China had the highest number of articles, followed by the United States, Taiwan, South Korea, Australia, and England, indicating that these countries are leaders in this field. China has already established a strong country-centered position and plays a significant role in mediating the global collaborative network. Conversely, the centrality of other countries was relatively low, indicating a lower level of influence and cooperation in most countries.

A total of 1274 institutions from 66 countries participated in the WoS literature analyzed in this study. The institution with the highest number of publications was the Shanghai University of Traditional Chinese Medicine (SUTCM), which published 42 articles. Most of these institutions were universities or hospitals related to TCM. Affiliated institutions were mainly hospitals or schools that were based or affiliated with the main institution. However, there was still no complete and interconnected system of cooperation between schools and organizations (**Figure 1D**). Next, we analyzed the institutions of the authors in the literature from the Chinese databases. As a result, it can be seen that most of the articles came from Chinese medicine colleges, of which the largest number of articles came from Guangzhou University of Traditional Chinese Medicine and Ningxia Medical University (**Supplementary Table 3**). This suggests that most clinical studies on acupuncture treatment for CRC were conducted in universities and colleges. Guangzhou, a region in China with a high degree of recognition of Chinese medicine, has a high level of acceptance among the people. Consequently, related studies have been conducted relatively smoothly and the results are convincing, leading to an increase in the number of studies. However, there is a lack of cross-unit collaborations and insufficient cross-regional communication and cooperation within China. The incidence of CRC is also related to geography and weather, which highlights the need for larger, cross-regional, and multiparty collaborative clinical studies in the future.

RETRACTED

### 3.4 Journal sources of literature analysis

Most articles in the WoS come from *Acupuncture in Medicine*, *Jama Surgery*, *Trials*, with *Jama Surgery* with an impact factor of 16.9. Furthermore, most journals sourced were in Q1, and the majority of impact factors ranged from 2.6 to 4.6. Moreover, the journal sources of the articles from the Chinese databases derived from the *Shanghai Journal of Acupuncture and Moxibustion*, *Chinese Acupuncture & Moxibustion*, *Journal of Sichuan of Traditional Chinese Medicine*, and *Acupuncture Research*. Among which those papers belonging to PUK and CSCD-C were *Chinese Acupuncture & Moxibustion* and *Acupuncture Research*, with impact factors of 2.509 and 2.756, respectively, and were the more authoritative journals in the field of acupuncture in China, and the quality of their published articles are all high. In general, this study indicated that the articles we included in the analysis were representative and that acupuncture was effective in the treatment of CRC (**Supplementary Table 4**).

### 3.5 Article citation analysis

The number of citations reflects the impact of the paper. If a paper is cited many times, it means that it has high recognition and influence in the field. In the literature reviewed for this study, a total of 1220 articles were cited. The most frequently cited articles were by Ng et al. (12) in the WoS database and by Zhang et al. (13) in the Chinese databases, both with over 120 citations. The article by Pu, C.-Y (14) was the second most cited in the WoS, with 38 citations followed by the article by Liu et al. (15) with 35 citations. In the Chinese databases, the study by Gui et al. (16) was cited 48 times and Li et al. (17) was cited 40 times. These findings suggest that these authors in this field had a strong specialization and significant impact (**Table 1**).

RETRACTED

**Table 1:** Table of count of article from WoS and Chinese databases.

databases	References	Title	Journal	Cited
Articles from WoS	Ng SSM et al. (12)	Electroacupuncture Reduces Duration of Postoperative Ileus After Laparoscopic Surgery for Colorectal Cancer	Gastroenterology	128
	Pu, C. -Y. et al.(14)	The determinants of traditional Chinese medicine and acupuncture utilization for cancer patients with simultaneous conventional treatment	Eur J Cancer Care (Engl)	38
	Liu Yihong et al. (15)	Acupuncture and Related Therapies for Treatment of Postoperative Ileus in Colorectal Cancer: A Systematic Review and Meta-Analysis of Randomized Controlled Trials	Evid Based Complement Alternat Med	35
	Hsieh Yueh-Ling et al. (18)	Laser acupuncture attenuates oxaliplatin-induced peripheral neuropathy in patients with gastrointestinal cancer: a pilot prospective cohort study	ACUPUNCTURE IN MEDICINE	34
	Deng, Gary et al. (19)	A Phase II, Randomized, Controlled Trial of Acupuncture for Reduction of Postcolectomy Ileus	Ann Surg Oncol	32
	Kim, Kun Hyung et al. (20)	Acupuncture for recovery after surgery in patients undergoing colorectal cancer resection: a systematic review and meta-analysis	Acupunct Med	29
	Li Hong-Ping et al. (21)	Electroacupuncture decreases Netrin-1-induced myelinated afferent fiber sprouting and neuropathic pain through μ-opioid receptors	J Pain Res	25
	Yeo Ji-Hee et al. (22)	Repetitive Acupuncture Point Treatment with Diluted Bee Venom Relieves Mechanical Allodynia and Restores Intraepidermal Nerve Fiber Loss in Oxaliplatin-Induced Neuropathic Mice	J Pain	23
	GUI Lin et al. (16)	The Acupuncture-moxibustion Treatment for Patients with Anterior Resection Syndrome After the Operation for Rectal Cancer	Liaoning Journal of Traditional Chinese Medicine	48
	LI Dongxiao et al. (17)	Effects of acupuncture therapy combined with nutrition support of enhanced	Guangxi Medical Journal	40
		recovery after surgery on colorectal cancer in perioperative period		
	GU Xuying et al. (23)	Effect of warm acupuncture on gastrointestinal response in patients undergoing postoperative abdominal heat infusion chemotherapy for colon cancer	Acupuncture Research	31
	LI Boping et al. (24)	Curative Effect Observation of Acupuncture Combined with Chinese Medicine in Treatment of Postoperative Gastrointestinal Dysfunction of Colorectal Cancer Patients	Progress in Modern Biomedicine	29
	LI Lin et al. (25)	Effect of Tongxiayao Recipe Combined with Acupuncture and Moxibustion on Delayed Diarrhea after Chemotherapy for Colon Cancer	Electronic Journal of Clinical Medical Literature	23
	SUN Hui et al. (26)	Effects of warm acupuncture and moxibustion on immune function and intestinal flora in patients with colorectal cancer after radical operation	Acupuncture Research	23
	LIANG Zunxiao et al. (27)	Effect of fast track surgery concept combined with acupuncture on gastrointestinal function recovery after colorectal cancer surgery	China Medical Herald	22

RETRACTED

### 3.6 Co-citation cluster analysis

In this study, we examined the citations of literature related to acupuncture for the treatment of CRC. Using clustering analysis, we identified the most highly referenced literature, or key nodes in WoS. Furthermore, we discussed the characteristics and research focus of acupuncture and related TCM in the treatment of CRC.

The significance and reasonableness of keyword clustering depend on the clustering modularity (Q value) and the clustering average profile value Silhouette (S value) (27). A Q value greater than 0.3 is considered significant for clustering structure, while an S value greater than 0.5 is considered reasonable and an S value greater than 0.7 is considered convincing. We set NodeType as CitedReference and TimeSlicing as 1993-2023 in CiteSpace to obtain the co-cited literature clustering mapping of acupuncture and related Chinese medicine therapies for colorectal cancer (**Figure 2**). The co-cited clustering map of literature on acupuncture and related Chinese medical therapies for colorectal cancer had 272 nodes, 753 connecting lines, 15 clusters, a network density of 0.0204, a Q value of 0.8973 (>0.3), and an S value of 0.9805 (>0.7).

**Figure 2:** Visualization of co-citation analysis from WoS.

According to the cluster mapping, “#1 Ic3”, with a total of 33 co-citations. The earliest co-citation in this cluster was published in 2007. “#2 spleen deficiency syndrome” has 31 co-citations, with the earliest co-citation in this cluster published in 2002. Cluster “#4 apoptoticeffects” has 21 co-citations, with the earliest co-citation in this cluster published in 2001. Cluster “#5 testicularmetastasis” has a total of 18 co-citations, with the earliest co-citation in this cluster published in 2007. Cluster “#9 cancerstemcells” has a total of 11 co-citation literature, with the earliest co-citation in this cluster published in 2009. Cluster “#10 cellproliferation” has a total of 18 co-citations, with the earliest co-citation in this cluster published in 2004. This result suggests that in the early 21st century, studies related to acupuncture for colorectal cancer began to explore the mechanism of action at the molecular level to evaluate its effects.

RETRACTED

### 3.7 Keyword Analysis

#### 3.7.1 Keyword co-occurrence

A higher frequency of keywords indicates a higher degree of research intensity, and a higher centrality indicates a higher degree of research importance (12). In this study, we performed a keyword visualization analysis to obtain a representative map. The WoS results showed that the key word “colorectal cancer” had the highest frequency of 182 cases, with a centrality of 0.48. Following “colorectal cancer,” “traditional Chinese medicine,” “acupuncture,” and “apoptosis” were all keywords with a centrality greater than 0.15, indicating their importance in the research (**Figure 3A**). In the same way, the result of Chinese databases indicated that “colorectal cancer” had the highest frequency of 32 occurrences, with a centrality of 0.83. The keywords “electroacupuncture” and “rectal cancer” had a centrality greater than 0.25, expressing their importance in the search (**Supplementary Table 5**). These findings suggest that the literature mainly focused on these keyword models. Additionally, comparing the data, it can be seen that acupuncture, warm acupuncture, chemotherapy, hot compresses, and acupuncture point therapy are commonly used in clinical practice to treat pain and diarrhea, urinary retention, tumor metastasis, and pain caused by CRC.

**Figure 3:** Keyword visualization and analysis mapping from WoS and Chinese databases. 电针: electroacupuncture; 揿针: intradermal acupuncture; 结肠癌: colon cancer; 免疫功能: immune function; 针刺疗法: acupuncture treatment; 针灸: acupuncture and moxibustion; 穴位: acupuncture point; 针刺: acupuncture; 直肠癌: rectal cancer; 胃肠功能: gastrointestinal function; 足三里: zu sanli (ST36); 肠癌术后: postoperative bowel cancer; 痛泻要方: tongxieyaofang Decoction; 预处理: pretreatment; 肠功能: intestinal dysfunction; 呕吐: vomiting; 腹腔镜: laparoscope. **(A)** Visualization of keyword frequency in WoS; **(B)** Visual analysis of keyword clustering in WoS; **(C)** Visual analysis of keyword clustering in a Chinese database; **(D)** Visual analysis of Burst words in WoS; **(E)** Visual analysis of Burst words in a Chinese database.

#### 3.7.2 Keyword clustering

Keyword clustering is a method that uses induction to group multiple keywords into a single tag, reflecting the hotspots in the research process. This approach helps to better focus on deciding future research directions (28). In the analysis of the WoS, the clustering produces 9 tags, sorted from 0 to 8, with smaller numbers indicating more keywords in the cluster. For example, “#0 acupuncture” “includes keywords such as acupuncture, chemotherapy, breast cancer, therapy, and quality of life.”#1 network pharmacology” includes keywords such as expression, cells and pathway. “#2 colon cancer” includes keywords such as apoptosis, traditional Chinese medicine, and colon cancer. “#3 colorectal cancer” includes CRC. **Figure 3B** shows that “#0 acupuncture” contains the most keywords, while “#8 neural regeneration” contains the least keywords. In the Chinese databases, producing 6 tags, sorted from 0 to 5. “#0 electroacupuncture” includes keywords such as electroacupuncture, intestinal function, preconditioning, traditional Chinese acupuncture, and Inflammatory response. “#1 intradermal needle” includes keywords such as CRC, intradermal needle, vomit and ST36. “#2 colon cancer” includes keywords such as colon cancer, electroacupuncture, and clinical observation (**Figure 3C**).

RETRACTED

In this visualization analysis, the Q value was 0.5831 (>0.3) and the S value was 0.7575 (>0.7), which can be considered significant and convincing for this clustering structure. Similarly, the Q value was 0.5214 (>0.3) and the S value was 0.8108 (>0.7) in Chinese databases, which are considered important and convincing.

#### 3.7.3 Burst words

Burst-word analysis is a useful tool for identifying the most significant keywords and recent research trends. This is crucial to summarize the themes of a research field and to predict future directions (29). In the study of the WoS, we generated a total of 229 emergent words, all of which appeared after the year 2012. The first emerging term was “natural products” in WoS, which appeared in 2012 and ended in 2014. In the period 2014 to 2018, we expected to see the emergence of terms such as “alternative medicine,” “management,” and “therapy,” The main keywords for the period 2017 to 2021 were “proliferation,” “modulation,” “*in vitro*,” “tumor growth,” and “mechanisms.” From 2019 to 2023, the keywords were “resistance,” “pathway,” “survival,” and “inflammation.” Among all emerging terms, “activation” was the most intense, with an intensity of 4.2 from 2013 to 2016 (**Figure 3D**).

In the Chinese databases, we generated a total of 126 emergent words, almost all appearing after the year 2010. The first emergent term was “acupuncture,” which appeared in 2010 and ended in 2015. From 2010 to 2014, the main keywords were “acupuncture,” “acupuncture points,” “rectal cancer,” “gastrointestinal function,” “ST36 (Zu san li),” “postoperative bowel cancer”, and “Tong xie yao prescription.” From 2017 to 2020, the main keywords included “bowel function,” “vomiting,” “laparoscopic,” “colon cancer,” “immune function,” and “acupuncture therapy.” Among all the emerging terms, “gastrointestinal function” was the most intense, with an intensity of 2.45 between 2011 and 2016 (**Figure 3E**).

RETRACTED

#### 3.7.4 Keyword clustering timeline

The timeline graph for keyword clustering studies the relationship between keywords and time based on keyword clustering. This graph reflects the trend of current hotspots over time (30). By analyzing the frequency and time of keyword appearance in different clusters, we can gain insight into the dynamics of the corresponding cluster labels on the time axis. Each node in the graph represents a release, and its position on the time axis indicates the corresponding release time. The density of the nodes at different time points reflects the dynamics of the corresponding cluster labels on the time axis. The cluster labels represent the topic of the study (31). The bigger the node, the brighter the color, which means that the keyword occurs more frequently and is hotter. In this analysis of WoS, there were nine clusters for the keywords: “#0 acupuncture,” “#1 network pharmacology,” “#2 colon cancer,” “#3 colorectal cancer,” “#4 inflammatory bowel diseases,” “#5 usnic acid,” “#6 integrative medicine,” “#7 estrogen receptor beta,” “#8 neural regeneration.” The keyword “colorectal cancer” in the cluster “#3 colorectal cancer” first appeared in 2000 and had the highest frequency. In Chinese databases, there were 6 clusters for the keywords: “#0 electroacupuncture,” “#1 intradermal needle,” “#2 colon cancer,” “#3 rectal cancer,” “#4 immune function,” “#5 acupuncture therapy.” The keyword “colorectal cancer” in the “#1 Intradermal needle” group first appeared in 2011 and had the highest frequency (**Figure 4**).

**Figure 4:** Keyword emergent word map and keyword timeline chart from WoS and Chinese databases. 电针: electroacupuncture; 揿针: intradermal acupuncture; 结肠癌: colon cancer; 免疫功能: immune function; 针刺疗法: acupuncture treatment. **(A)** Visualization of Keyword Clustering Timeline in WoS; **(B)** Visualization and Analysis of Keyword Clustering Timeline in Chinese Databases.

## 4 Discussion

This study used CiteSpace for the first time to investigate the current state of research on acupuncture, alone or in combination with other traditional Chinese medicine therapies for the treatment of CRC, and to identify current focus areas and future research directions. A total of 450 papers related to this topic were collected from the WoS and the Chinese databases between 1 January 1993 and 30 July 2023, and the growth trend of this research field has fluctuated over time. We retrieved 355 articles, which were contributed by 2462 authors. Li Q published the highest number of papers (32, 33), but the research mainly focused on the therapeutic study of acupuncture combined with Chinese herbs in CRC in mice. Therefore, this author was not the author most closely related to the topic of our study. In the era of globalization and online medicine, it is essential to have cross-cultural collaboration and communication. Institutions and individual researchers should focus on integrating resources, promoting international exchanges and cooperation, and leveraging the unique strengths of each country to advance the field and establish a new era of international cooperation.

RETRACTED

To date, 66 countries have published articles regarding acupuncture in the WoS. China leads the way with 285 published articles (80.28%), followed by the United States, Taiwan, South Korea, and Australia. As the birthplace of acupuncture, China has made significant progress in this field. However, most studies on CRC have focused primarily on its clinical efficacy, and the mechanisms of acupuncture for the treatment of CRC complications are poorly understood. Therefore, there is a pressing need to conduct numerous original studies to examine the current situation of acupuncture, alone or in combination with other TCM therapies, to treat CRC and its complications. These studies will offer empirical references for the specific directions of future research.

Most published articles were from higher education academic institutions in WoS and Chinese databases. A total of 1385 institutions published relevant articles, with the top five located in China from WoS: Shanghai University of Traditional Chinese Medicine (SUTCM), Nanjing University of Traditional Chinese Medicine (NUTCM), Guangzhou University of Traditional Chinese Medicine (GUTCM), Beijing University of Traditional Chinese Medicine (BUTCM), and China Medical University (CMU) in Taiwan, and with the top five located in China from in Chinese databases: Guangzhou University of Chinese Medicine, Ningxia Medical University, General Hospital of Ningxia Medical University, Nanjing University of Chinese Medicine, and Shandong University of Traditional Chinese Medicine. This indicates that Chinese institutions make significant contributions in terms of both absolute and relative influence. As the quality of medical care is closely related to the pace of economic development, the agency distribution table assists researchers in identifying and selecting appropriate partner institutions.

RETRACTED

Most clinical studies on acupuncture for CRC were published in highly influential journals. This study included a total of 217 journals, such as *Jama Surgery*, *Neural Regeneration Research*, *Supportive Care in Cancer*, and *Toxins* in WoS, as well as *Chinese Acupuncture and Moxibustion* and *Acupuncture Research* in Chinese databases. These journals are known for their high prestige and academic level. The fact that articles on acupuncture for CRC were published in such high-profile journals indicates that the clinical studies are of high quality and representative. This also helps to promote and popularize acupuncture for CRC.

This study revealed that the article with the highest number of citations in the WoS was published in *Gastroenterology*, with 128 citations. Similarly, the most cited article in CNKI was published in the *Chinese Acupuncture & Moxibustion* and had 120 citations. Most of the other highly cited articles were only cited between 20–40 times. This indicates that reading these articles can provide valuable insights into the current state of research in the field and can deepen the understanding of research trends and future directions and broaden research horizons and stimulate new ideas.

Keywords are crucial to reflecting a topic with both precision and generalization. During the analysis process, commonly used keywords were identified to pinpoint hotspots in the research field. Through co-occurring keywords and cluster analysis, it was found that there is a growing interest in using acupuncture and other TCM therapies to treat CRC, with an increasing degree of innovation both in WoS and Chinese databases. The keywords “colorectal cancer,” “traditional Chinese medicine,” and “acupuncture” had the highest centrality indexes, indicating that our selection of selection of literature was highly relevant to the research topic. The terms “colorectal cancer,” “apoptosis,” and “traditional Chinese medicine” have been observed to be the most frequently mentioned, indicating that the study of the role of apoptosis in the treatment of CRC with traditional Chinese medicine is gaining favor. “Immunologic function” and “gastrointestinal function” were high-frequency keywords in the Chinese databases, suggesting that acupuncture treatment of CRC is mainly related to the regulation of immune function and gastrointestinal function. This suggests that the current approach to treating CRC with TCM is increasingly focused on understanding the role of apoptosis, immune function, and gastrointestinal function, which will help in the future development and prediction of TCM mechanisms to treat CRC.

RETRACTED

As we can see from the timing of the keywords, acupuncture was initially used to treat CRC, but gradually evolved into a method to inhibit complications or resistance to chemotherapy drugs. In the process, basic experimental methods were used to explore the relevant mechanisms. In addition, “inflammation” and “immune function” were identified as important keywords related to the mechanism. This suggests that acupuncture can inhibit tumors or alleviate their complications and may be related to modulation of inflammatory and immune responses. These findings are consistent with the literature (34, 35), which suggests that exploring the mechanism of acupuncture or related combinations of Chinese medicines in the treatment of CRC has been fruitful. Further, this combination acts as a focal point in the research field of acupuncture for CRC and can be used as a direction for future prediction.

In terms of the timeline of appearance of keywords, the “acupuncture” cluster has the most keywords, while “colorectal cancer” has the highest frequency, centrality index, and the earliest appearance time. The distribution of keywords in the timeline and the density of different time nodes reflect the dynamic changes of the corresponding cluster labels and the focus of this study. The focus has shifted from clinical efficacy and theoretical analysis to research at the cellular level of the mechanism of action.

Acupuncture, alone or in combination with related TCM treatments, has shown remarkable results in the treatment of CRC over the past two decades. Its low toxicity and cost are among its advantages. To further improve the fundamental treatment of CRC and reduce mortality, recurrence, and morbidity, it is necessary to deepen our understanding of its mechanism of action and to research more efficient and optimized treatment plans. However, research on its mechanism of action is still in its infancy and requires a large number of cases, experiments, and analyses to be completed.

The information gathered from the WoS and Chinese databases on hot topics, co-cited literature, countries, institution author collaborations, journal source, and frequency of citations on acupuncture or related TCM treatments for patients with CRC encompassed most of the literature on the subject. Data analysis was impartial and relevant to the topic, providing information on the historical and current status of acupuncture or related TCM treatments for CRC patients. Additionally, CiteSpace was used to forecast future research prospects and directions. However, there are still obvious limitations to this topic. Due to the constraints of the CiteSpace software on data format, we can only analyze data from the WoS database, which may result in data bias and did not fully reflect all available literature. Additionally, our selection of only the published literature in English may also lead to bias in visualization analysis.

RETRACTED

## 5 Conclusions

Using CiteSpace software, this study provides evidence of collaborative communication between authors, countries, and institutions. Although we included studies from both the WoS and Chinese databases, the results were found to be similar in terms of the number of publications, journals, and citations. Therefore, this study suggests that current research trends are primarily focused on the clinical efficacy of acupuncture and other Chinese medicines in treating CRC, as well as the efficacy and mechanism of acupuncture and other Chinese medicines in treating CRC in mice. It is important to further investigate the therapeutic mechanisms of acupuncture and other TCM combinations for CRC. This will allow the development of more in-depth and efficient treatments based on optimal therapeutic regimens tailored to individual patients.

In recent years, there has been a growing interest in using Chinese herbs and acupuncture as treatments for CRC. In addition, several studies have investigated the effectiveness of combining acupuncture and herbal medicine to develop more efficient treatment methods. However, greater collaboration and systematic exchanges among research institutions are needed. Current research in this field is focused on the fact that acupuncture, alone or in combination with other Chinese medicine therapies, has shown significant efficacy in treating CRC and its complications. The main mechanism of action is related to inflammation and immunoregulation. Furthermore, the growing number of research studies on acupuncture and TCM indicates that their therapeutic effects are increasingly recognized in clinical practice.

## Data availability statement

The raw data supporting the conclusions of this article will be made available by the authors, without undue reservation.

## Author contributions

LZ: Data curation, Formal analysis, Writing – original draft. XQ: Data curation, Formal analysis, Investigation, Software, Writing – original draft. LS: Data curation, Software, Writing – original draft. CW: Data curation, Formal Analysis, Investigation, Software, Writing – review & editing. XN: Project administration, Resources, Supervision, Writing – review & editing. QF: Conceptualization, Methodology, Resources, Supervision, Validation, Writing – review & editing.

## Supplementary material

Supplementary Table 1 Table of count of article from WoS and Chinese databases.

RETRACTED

Supplementary Table 2 Top 44 authors in the number of published articles from WoS and Chinese databases.

Supplementary Table 3 Top 13 Sources in terms of publications from Chinese databases.

Supplementary Table 4 Top 21 authors from WoS and Chinese databases. KMCT, The key magazine of China technology; PKU, Keking University Journals Platform; CSCD-E, Chinese Science Citation Database Expanded; CSCD-C, Chinese Science Citation Database Core.

Supplementary Table 5 Keywords with high frequency of occurrence from WoS and Chinese databases.
